The article "Meta-Analysis of Mechanism of Influence of CRY2 on the Differentiation of Mouse Osteoblast through the Regulation of Wnt/Β-Catenin Signaling Pathway" was retracted in 2024. Reasons: signs of a paper mill; suspected computer-generated content; unreliable results or conclusions; concerns about the data.

# Meta-Analysis of Mechanism of Influence of CRY2 on the Differentiation of Mouse Osteoblast through the Regulation of Wnt/*Β*-Catenin Signaling Pathway

**DOI:** 10.1155/2022/3727165

**Published:** 2022-08-21

**Authors:** Chao Ma, Chaojian Yang, Tong Xie, Wenjuan Dai, Jun Ma

**Affiliations:** ^1^People's Hospital of Ningxia Hui Autonomous Region, Yinchuan, Ningxia, China; ^2^Ningxia Medical University, Yinchuan, Ningxia, China

## Abstract

Noncoding RNAs were discovered to control a variety of developmental mechanisms, including osteogenesis. According to emerging evidence, cryptochrome circadian-regulating (CRY) proteins have emerged as essential controllers of osteoblast differentiation. The linked processes, on the other hand, are still unknown. The specific process that underpins osteoblast differentiation and proliferation is yet unknown. This research gives a meta-analysis of CRY2's impact on mouse osteoblast differentiation via the control of the WNT/*β*–catenin signaling pathways. Western blot and quantitative real-time PCR were used to identify Cry2 expression levels, components in the osteoblast-associated signaling pathway, and osteoblast transcription markers. The osteogenic condition was measured utilizing alkaline phosphatase (ALP) and alizarin red (AR) staining, whereas cell growth rates were measured using CCK8 assays. An ectopic bone formation experiment was used to determine the osteogenic potential of osteoblasts. Cry2 stimulates the osteogenic development of mouse osteoblasts through canonical Wnt/*β*-catenin signaling, according to the findings.

## 1. Introduction

To maintain bone metabolic balance, osteoblasts are required for bone synthesis, which is followed by osteoclast-mediated bone resorption. Proliferation and differentiation help with osteogenesis. MSCs and osteoblasts are good candidates for bone regeneration because of their ability to manufacture, secrete, and mineralize bone matrix. To see whether sexual dimorphism altered its reactions to systematic hormones during implant osseointegration, researchers employed microstructured Ti implants encapsulating osteoblast [1]. The expressions of regulatory genes, osteoblast differentiation indicator genes, signaling pathways, and mineral accumulation are all involved in osteoblast differentiation. It is critical to ensure appropriate control of osteoblast production as a portion of the bone regeneration mechanism, which maintains the bone strong. While bone growth is not properly controlled, numerous clinical disorders appear. At various phases of osteoblast differentiation, distinct signaling pathways and elements are adopted. For example, the Indian hedgehog (Ihh) (The Indian Hedge Hog (Ihh) gene family produces three signaling molecules. The Hh family of genes, including Sonic Hedge Hog (Shh), Desert Hedge Hog (Dhh), and Ihh, control a variety of fetal developmental processes. During the development of limbs, the Ihh homolog plays a role in the production of chondrocytes) increases the differentiation of mesenchymal progenitor tissues during endochondral bone growth. Notch signaling (A single-pass transmembrane receptor protein, the notch receptor. It is a hetero-oligomer made up of a big extracellular section that interacts with a smaller piece of notch protein made up of a short extracellular area, a single transmembrane-pass, and a small intracellular region in a calcium-dependent, noncovalent contact) enhances the development of preosteoblasts into osteoblasts but inhibits the production of preosteoblasts in MSCs. WNT canonical and noncanonical pathways are critical for membranous and endochondral bone growth [2]. Osteoblast differentiation is influenced by osteoclast, MSC, and adipocyte proliferation in earlier studies. Coculture of osteoblasts with these cells, for instance, could replicate in vivo conditions to study their interactions via secreted cytokines and autocrine and paracrine elements. To ensure that bone synthesis influenced osteoblast differentiation, several chemicals were created during bone resorption.

MSCs limit osteoblast development in osteogenic-inducing conditions. As a result, it is important to understand the interaction between osteoblasts and other cells, as well as the elements that influence bone production [3]. A membrane-bound bone deposition is a mechanism that produces osteoblast from MSCs. Collagen (COL), osteocalcin (OC), proteoglycan, and unmineralized biological components like osteoblasts are all secreted by them. Osteoclasts, on the other hand, are formed from hematopoietic stem cells and help in bone growth as well as calcium generation as a byproduct. The osteocytes are mature osteoblasts that have been integrated into the bone matrix and maintain the shape of the bone. Osteoporosis, Paget's disease (A persistent bone ailment known as Paget disease. It enlarges and deforms the bones. Excessive breakdown and distortion of bone can lead it to become dense but brittle. In adults over the age of 50, the condition is the second most frequent bone disorder after osteoporosis), rickets (Rickets is an illness in which your child's bones become overly soft, leading them to distort, bend, and break more easily. Rickets is not the same as adult-onset osteomalacia. The distinction between the two is that rickets mainly affects youngsters since their bones are still growing, resulting in bowed or bent bones), and other musculoskeletal illnesses like (Carpal tunnel syndrome is a type of carpal tunnel syndrome that affects the (CTS), injuries to the back and discomfort in the back arthritis, ergonomics, workplace controls, and development and implementation) can be caused by an imbalance in the activities of osteoblast and osteoclast. Osteogenesis is a sequence of events rather than a single event, whereby tissues multiply, develop, and diversify from preosteoblasts to immature osteoblasts and then to matured osteoblasts. Several signaling pathways and interactions of transcriptional regulators contribute to promoting cell differentiation by controlling the expressions of downstream osteogenic genes during such phases of differentiation [4].

Osteoblasts play an important role in bone formation, ossification, and fracture repair. Osteoblasts are responsible for both repairing the small fissures that occur as a result of regular use and contributing to the dynamic qualities of bone. MSC releases a diverse spectrum of bioactive chemicals that aid in the creation of an ideal regeneration environment. This area is advancing quickly, with the possibility to be utilized in medical settings [5]. Osteoblast differentiation is influenced by osteoclasts, MSCs, and adipocyte differentiation in earlier studies. Coculturing osteoblasts with all of these difficulties, for example, might mimic an in vivo condition and allow researchers to investigate interactions via secreted cytokines, as well as autocrine and paracrine components. To ensure that bone production influenced osteoblast differentiation, several chemicals were created during a bone turnover. Under osteogenic-inducing circumstances, MSCs suppress osteoblastic activity. As a result, it is important to understand the interaction between osteoblasts and other tissues, as well as the elements that influence bone production [6].

This paper analyzes the mechanism of influence of CRY2 on the differentiation of mouse osteoblasts through the control of WNT/*β*-catenin signaling pathways. The further part of the paper is structured as follows: part II provides the related literary works and problem statement. Part III explains the methodology used in this study. Part IV analyzes the performance of the methodology used. And, finally, part V concludes the concept used in the paper.

## 2. Related Works

Zhang et al. [7] examined the expressions of the N6-adenosine methyltransferase METTL3 and discovered that it was upregulated at the time of osteoblast differentiation and downregulated following lipopolysaccharide (LPS) stimulation. In LPS-induced inflammation, they suppressed METTL3 and found lower concentrations of osteogenic biomarkers, alkaline phosphatase (ALP) activities, calcified components, and also, Smad1/5/9 phosphorylation. The same regulatory mechanism was observed while the m6A-binding protein YTHDF2 was suppressed: METTL3 reduction increased the micro-RNA expressions and integrity of negative controllers of Smad signaling. Furthermore, METTL3 reduction elevated phosphorylation, which boosted proinflammatory cytokine production. After using MAPK signaling inhibitors, the rise in cytokines production was stopped. CRY2 reduction facilitated osteoblast differentiation, according to Tang et al. [8]. Runt-associated transcriptional factor 2 (Runx2), ALP, osteocalcin (OCN), and osteopontin (OPN) expressions are all significantly suppressed. miR-7-5p which was substantially increased during osteoblast development was found to be precisely targeting CRY2. Upregulation of miR-7-5p and promotion of osteoblast differentiation induce the levels of transcriptional factors. Furthermore, miR-7-5p was stimulated by the signal transducers and activators of STAT3 to greatly increase the expressions of the osteogenesis genetic markers and mineral production. Rev-erbs inhibit the development of osteoclasts and osteoblasts, according to Kim et al. [9]. The findings show that Rev-erbs play a role in bone remodeling on a molecular level, and they give a biological basis for a possible therapeutic approach for treating a bone disease associated with excess bone resorption. The Rev-Erb proteins belong to the nuclear receptor (NR) group of intracellular transcription factors and are important clock regulators. Rev-Erb alpha and Rev-Erb beta are two types of the receptor, each expressed by a different gene (NR1D1 and NR1D2, respectively). Hirai [10] revealed the expression of sympathetic nervous system-regulated clock genes as well as clock-controlled genes, which influence bone formation. In osteoblasts, adrenergic receptor (AR) signaling seems to control cellular performance by regulating the production of clock genes, which regulate the circadian rhythm. Karsenty [11] proposed that the transcriptional component that is a differentiation component for a specific tissue type must be expressed in progenitors of that tissue type, govern the expressions of every cell-specific gene in that tissue type, stimulate expressions of the above genes while aberrantly conveyed in alternate kinds of cells, and be required for such cell differentiation in vivo, in mice, and humans. The transcriptional component now regarded as the primary gene of osteoblast differentiation, as outlined in this article, is among the few differentiation elements that meet all of these requirements. Takarada et al. [12] demonstrated that the clock system modulates bone regeneration and mass through its activation in bone-forming osteoblasts. The findings imply that the osteoblastic clock system regulates bone regeneration and mass at a complex level via a process associated with the control of 1,25 (OH)_2_D_3_-induced Rankl production in osteoblasts. Progressive and environmental factors influence the transcription activity of osteoblast at multiple phases, from lineage devotion through differentiation, with the engagement of coelements, mRNAs, epigenetics, systematic components, circadian rhythms, and the microenvironment. These concerns are discussed regarding transcriptional regulation in osteogenesis by Chan et al. [13]. Peng et al. [14] investigated how Cry1 affects the multiplication and differentiation of bone marrow MSCs (BMSCs) produced by low-level laser irradiation (LLLI). BMSCs reacted to LLLI therapy (660 nm; 10 mW) in a dosage- and time-reliant way, according to the findings. Cry1 depletion reduced cell survival, multiplication, and the transcription of cell cycle progression. The data showed that forcing Cry1 transcription boosts BMSC susceptibility to LLLI, implying that induced Cry1 transcription is a unique technique for enhancing MSC-based treatment in clinics. Zheng et al. [15] used lentiviral and adenoviral vectors to mute or upregulate BMAL1 or Per2 in BMSCs and then used MTT, flow cytometry, RT-qPCR, Western blotting, and ChIP-Seq studies to figure out what was going on. Bmal1 and Per2 had a synergic activity on BMSC multiplication and differentiation, according to the findings. BMAL1 and Per2 also blocked the WNT/*β*-catenin signaling pathway that was followed by downregulation of Ror expression and overexpression of Rev-erb expression, both of which were important components of circadian clock genes (CCGs). It could be the process through which BMAL1 and Per2 prevent BMSCs from undergoing osteogenic differentiation. Luo et al. [16] evaluated the administration of CCG in osteoblasts or osteoclasts, as well as the energy metabolism of bones and the connection between the circadian clock, bone regeneration, and energy metabolism. They also talked about the therapeutic value of modifying energy metabolism or controlling circadian clocks on bone formation and repair. Min and Jang [17] explored the role of Per1 in osteoblast differentiation. Bone morphogenetic proteins 2 (BMP2) was used to induce osteoblastic development in MC3T3-E1 cells. RT q-PCR was employed to assess the activity of the osteogenic marker gene and Per1 mRNA. BMP2 therapy enhanced Per1 mRNA expressions in MC3T3-E1 tissues, which was unexpected. The impacts of electromagnetic wave stimulation (EMS) on osteoblast multiplication and differentiation were studied by Pauly [18]. The impacts of several EMS treatments on multiplication, alkaline phosphatase (ALP) activity, and mineral accumulation were studied utilizing primary neonatal calvaria osteoblast-lineage cells. Wu et al. [19] reviewed previous research on the role of the circadian rhythm in bone homeostasis and disease. A key purpose of this study is to see how the circadian cycle affects osteoblast performance, osteoclast activity, and osteoblast-osteoclast interaction. They intended to gain a finer knowledge of the circadian rhythm in bone metabolism, as well as fresh perspectives into the control and therapy of bone diseases including osteoporosis. Tsang et al. [20] used the mouse with conditional elimination of BMAL1 in osteoclast and mesenchymal tissues of the limbs to analyze the role of the circadian molecular clock in various bone cell kinds. Employing a lentiviral vector containing RNAi series, Zhuo et al. [21] reduced Bmal1 transcription in bone marrow-derived MSCs (BMSCs), increasing the osteogenic differentiation potential of BMSCs. Maria and Witt-Enderby [22] characterized clock gene expressions and functions in bone, as well as how its rhythm affects osteoblasts and osteoclasts' activities and differentiation, as well as bone metabolism; they further addressed factors, which cause circadian interruption of bone rhythms, as well as methods of managing healthier bones in a society that improves it. Li et al. [23] identified and demonstrated the involvement of cholesterol-25-hydroxylase (CH25H) in stem cell development, as well as investigated the process. According to Karvande et al. [24], parathyroid hormone (PTH) increases osteoblast differentiation by promoting glucose-dependent miR-451a production. The data showed that increased osteoblast differentiation and bone growth in the presence of PTH medication is a result of increased miR-451a concentrations mediated by glucose metabolism. As a result, this miRNA can be used as a targeted therapy for bone loss. Yin et al. [25] used an mRNA/lncRNA microarray paired with gene coexpression assessment to identify osteogenic lncRNAs. In vitro and in vivo examinations were conducted on the selected lncRNAs to determine their biological purpose. The lncRNA's impact on osteogenic transcriptional regulators was also investigated. Paine et al. [26] used microcomputed tomography and histomorphometry to assess variations in bone morphology and total bone architecture in wild-type and Thy1 knockout mice's lengthy bones. Bao et al. [27] investigated the impact of osteoblast CA-*β*-catenin on bone qualities. According to von Kossa staining and sirius red staining, CA-*β*-catenin animals had decreased mineralization rates and disordered collagen in lengthy bones. CA-*β*-catenin mice also had lower bone density. The impact of CA-*β*-catenin on the biochemical processes of osteoblast was then explored, and it was discovered that expression degrees of osteocalcin, an indicator for delayed osteoblast differentiation, were reduced in CA-*β*-catenin mice, whereas expression degrees of osterix and ALP, two indicators for earlier osteoblast differentiation, enhanced.

### 2.1. Problem Statement

Primary mouse osteoblasts are still appropriate tissues for simulating internal procedures, particularly in genetically engineered animals. At various stages, endogenous (Cytokines are multifunctional molecules that mediate a variety of pathological processes. Investigators learned a lot about cytokines when they investigated them as endogenous mediators of fever long before they were discovered as immune system growth factors or bone marrow stimulants) and exogenous cytokines (Exogenous cytokines improve macrophage survival in organ grown embryonic rat tissues. Background information: macrophage precursors can be found in embryonic rats shortly after hematopoiesis begins), as well as micro RNAs, play an important role and address specific genes. The surface morphology of Ti discs was shown to stimulate differentiation of osteoblasts of less matured tissues. As a result, it is crucial to understand the phenotypic maker's expression profile at distinct phases of osteoblast differentiation. The techniques of initial osteoblast differentiation have been detailed in previous articles. Nevertheless, numerous issues remain, like contamination of other cells such as fibroblasts, chondrocytes, and osteocytes. It is unknown whether this method is suitable for rats or what differences exist in gene expression and mineralization capabilities between rat and mouse osteoblasts.

## 3. Materials and Methods

Osteoblasts are cells that specialize in the synthesis and mineralization of extracellular matrix. In mice, osteoblasts, and osteoclasts, which are bone-resorbing tissues, work together to maintain bone homeostasis. Osteoblast formation and bone remodeling are controlled by a coordinated interaction between osteoblasts and osteoclasts. To govern both the production and preservation of bones, osteoblast development necessitates a large number of transcriptional regulators (Transcriptional regulation is the mechanism through which a cell controls the conversion of DNA to RNA (transcription) and hence orchestrates gene activity). MSC-derived osteoblasts make up 5% of bone tissues and are essential for the formation of type I collagen and the deposition of calcified nodules, which aids bone growth. The CRY2 is a critical element of the circadian clock that is required for the construction and preservation of circadian rhythms. CRY2 is a transcription inhibitor that inhibits the transcription of genes and is linked to a variety of physiological functions. According to a rising number of studies, the circadian rhythm may regulate specific osteogenic differentiation. Cry2-/- animals, for example, had a considerable increase in bone density at the age of 12 weeks. Furthermore, the expression of peroxisome proliferator-activated receptor d (PPARd) genes was elevated in the Cry2-/- animal's myotubes and muscles, enhancing osteoblast development via the sirtuin 1-dependent signaling pathway. On the other hand, CRY2's specific strategy is unknown. In this section, the methodology used for the mouse osteoblast differentiation using CRY2 is discussed. The schematic portrayal of the suggested method is depicted in Figure 1.

### 3.1. Reagents and Drug Preparation

Sigma-Aldrich provided Dexamethasone, Ascorbic acid, -Glycerophosphate, and alizarin red S. Dexamethasone stock solutions are diluted in dimethyl sulfoxide (DMSO), whereas ascorbic acid and -glycerophosphate are diluted in phosphate-buffered saline (PBS) at concentrations of 1 mM, 10 mM, and 1 M, correspondingly, and held at 20°C before being dissolved in growing media just before osteogenic induction procedures. PBS is used to dissolve AR-S at a dosage of 40 mM. KY1220 is a WNT/*β*-catenin specific inhibitor purchased from MedChem Express that was synthesized in DMSO at a dose of 10 mM, kept at 80°C, and used at a dose of 25 *μ*M.

### 3.2. Cell Culture and Osteogenic Induction

Cell lines such as C3H10, C2C12, and 293T were bought from ATCC and grown in Dulbecco's Modified Eagle Medium (DMEM) provided with 10% fetal bovine serum (The liquid portion left after the blood was collected from a bovine fetus coagulates is known as foetal bovine serum (FBS). To make serum, cells, coagulation fibrinogens, and proteins are removed by centrifugation). Differentiation of osteoblasts was stimulated using osteogenic media comprising 50 *μ*g/mL of ascorbic acid, 10 mM *β*-glycerophosphate, and 1 mM dexamethasone, which was replenished every two days. The samples were incubated at 37°C in a humid environment with 5% carbon dioxide.

### 3.3. Construction of Plasmid

LncBio (Shanghai) provided micro-RNA and antimicro-RNA precursor cultures of miR-7-5p (The mir-7 microRNA precursor is represented by this family. A wide variety of animals have had this miRNA predicted or experimentally confirmed. miRNAs are transcribed as 70 nucleotide precursors which are then processed by the Dicer enzyme into a 22 nucleotide product. The mature sequence in this example is derived from the 5′ arm of the precursor) and antimiR-7-5p in lentiviral vectors, as well as lentiviral plasmids. Three plasmids are included in the lentivirus system for shRNA expression. Addgene System Biosciences (SBI) provided the lentiviral vector pCDHCMV-MCS-EF1-puro. Two shRNAs addressing the mouse CRY2 mRNA series were introduced into the lentiviral vector pLKO.1-puro, as per previously published procedures, to knock down CYR2 expression. A complete-length coding DNA series of mouse CRY2 was expanded utilizing forward primer 5′-GCTCTAGAATGGCGGCGGCTGCTGGTGGCAG-3′ and the reverse primer with hemagglutinin (HA) tag: 5′CAAGGAAAAGCGGCCGCTCAAGCGTAATCTGGAACATCGTAATCTGGAACATCGTAATCTGGAACATCGTAATCTGGAACATCGTAATGTGGAACATCGTAATCTGGAA.

### 3.4. ALP Staining and Alizarin Red (AR) Staining

As per the literature, osteogenic stimulation of cells can result in the production of calcified nodules and calcium accumulations, which can be detected by AR staining; hence, we used alizarin red staining in this investigation. The samples were treated with 4 percent paraformaldehyde and then cleansed 3 times with onetime phosphate-buffered saline to eliminate the paraformaldehyde. The cells were further treated for 1 hour at 37°C with a 40 mM AR dye solution to mark the calcium deposits. Thereafter, every one of the plates was examined after being cleaned with deionized water to remove any unconjugated AR. The Leagene ALP Kit was used to stain the alkaline phosphatase. The samples were cleaned in PBS and incubated in four percent paraformaldehyde for 30 mins at room temperatures before being stained. Plates with labeled tissues were observed. The AR staining was measured by dissolving stained tissues in 10 percent cetylpyridinium chloride and measuring the retrieved solution's absorption at 562 nm.

### 3.5. Alkaline Phosphatase Activity Assay

Samples were tested for ALP activity after osteogenic induction utilizing a commercial kit and following the production guidelines. The protein level was estimated utilizing the bicinchoninic acid (BCA) technique. The comparative alkaline phosphatase activity was then adjusted to overall protein content using conventional methods. The ALP staining was quantified by dissolving stained tissues in 10 percent (*w*/*v*) cetylpyridinium chloride and measuring the retrieved solution's absorbance at 562 nm.

### 3.6. CCK-8 Assay

The CCK-8 toolkit was used to test the impact of CRY2 on C3H10 and C2C12 tissue growth. Three replicates of C3H10 and C2C12 tissues were digested and seeded at 3∗10^3^ and 1.5∗10^3^ cells per well, correspondingly, into 96-well plates. After culturing for 0, 24, 48, 72, and 96 hours, 10 liters of CCK-8 reagent were combined with 100 liters of new medium and poured into every well. The plates were then incubated at 37°C for 2 hours, and the absorption of 450 nm was measured using a Tecan Infinity 200Pro multiwell plate reader. The testing was performed 3 times.

### 3.7. In Vivo Ectopic Bone Formation Assay

To determine if CRY2 overexpression increases osteoblast differentiation in vivo, an ectopic bone formation test was used. Female BALB/c naked mice aged four weeks had 2∗10^6^ regulation tissues or CRY2-upregulated C3H10 tissues administered subcutaneously into the skin under the left front leg. Each group was given seven duplicates. The transplants were retrieved and treated in ten percent formaldehyde for HE, Masson's staining, and immunohistochemistry (IHC) of osteocalcin (OCN) to assess osteogenesis after 6 weeks of monitoring. All animal care and research methodologies were following China's Animal Management Guidelines and were authorized by approved by People's Hospital of Ningxia Hui Autonomous Region's ethical committee.

### 3.8. Real-Time Reverse Transcription PCR

The TRIzol reagent was employed to separate overall RNA from cultivated cultures as per the manufacturer's guidelines. The Applied Biosystems 7500 Real-Time PCR Systems were employed to perform real-time PCR. Overall RNA was reversely converted into cDNA utilizing the TransScript microRNA. Real-time PCR evaluation was done utilizing the FastStart Universal SYBR Green Master to identify miRNA concentrations. The miRNA test utilized U6 as an internal reference, and the procedures were performed in triplicate. To assess the fold variation in expressions between the experiment and control groups, the 2-technique was used to estimate proportional mRNA or miRNA levels of expression.

### 3.9. Western Blotting

The radio immune precipitation assay (RIPA) lysis buffer comprising the protease inhibitor cocktail was used to lyse the tissues. The BCA Protein Assay Kit was used to assess the protein content. 10 percent SDS-PAGE was used to isolate equivalent quantities of protein, which were then transported to PVDF membranes. After blockage, membrane-bound proteins were provided with fundamental antibodies overnight at 4°C. Protein concentrations were assessed employing improved chemiluminescence reagents after cleaning and incubation with secondary antibodies. Proteintech provided the main CRY2 antibodies. Santa Cruz provided the p-STAT3 (S727) and P300 antibodies. Abcam provided the OPN and CLOCK antibodies. Sigma-Aldrich provided the beta-actin antibody. All of the trials were carried out three times. Between 5 s and 2 minutes, all blots are revealed for visualization.

## 4. Results and Discussion

In this section, we will discuss the suppression of CRY2 improves osteoblast differentiation, CRY2 is a direct target of miR-7-5p, the impact of CRY2 upregulation on bone formation in vivo, and upregulation of the CRY2 activated the canonical WNT/*β*-catenin signaling pathway in detail.

### 4.1. Suppression of CRY2 Improves Osteoblast Differentiation

We used short hairpin RNAs (hRNAs) to suppress the natural expressions of CRY2 in C3H10 and C2C12 tissue cultures to clarify the impact of CRY2, a transcription inhibitor, and a significant part of the circadian clock, which might show a vital part in the differentiation of osteoblasts. CRY2 protein expression is effectively reduced by CRY2 shRNA when contrasted to control shRNAs (Figure 2). After suppressing CRY2, we performed RT-qPCR to assess the degrees of expression of osteoblast differentiation indicators. Following knocking down CRY2 expression, the expression of numerous bone-specific indicators increased (Figures 3(a) and 3(b)).

We also investigated how CRY2 affects osteogenic differentiation and calcification. In the osteogenic induction medium, tissues representing shRNA control and CRY2 shRNA were grown. Calcified nodules are stained red with alizarin red staining following 21 days of osteogenic induction, as can be seen in (Figures 4, 5(a), and 5(b)). In CRY2 shRNA consistently transfected cells, AR staining and ALP staining were compared to the control group cells.

CRY2 knockdown hampered the development of mineralized aggregates when stained with alizarin red. Likewise, when CRY2 shRNA-treated tissues were contrasted to control samples, ALP staining and activity were much higher (Figures 4, 5, 6(a), and 6(b)). Such findings indicate that CRY2 inhibits osteogenic differentiation.

### 4.2. CRY2 Is a Direct Target of miR-7-5p

We utilized TargetScan, miRWalk, microrna.org, and miRDB to identify the probable microRNAs, which may address the 30 UTR of CRY2 microRNA to examine the biochemical pathway of CRY2-associated osteogenic differentiation. We chose 11 potential miRNAs, but it was discovered that CRY2 expression was only reduced following miR-7-5p upregulation at the mRNA degree (Figure 7). The expression of osteocalcin was reduced after CRY2 upregulation. Upregulation of miR-7-5p, on the other hand, restored the suppression of osteoblast differentiation caused by upregulation of CRY2 (Figure 8). All of the evidence suggests that CRY2 is a miR-7-5p downstream target.

### 4.3. The Impact of CRY2 Upregulation on Bone Formation In Vivo

We used animal experiments using control and CRY2 overexpressing C3H10 and C2C12 cells to verify the ex vivo findings. In both groups, 7 nude mice were placed live, and ectopic bone growth was observed.

HE staining revealed that C3H10 and C2C12 cells in the CRY2-cDNA group generated more bone-like structures than those in the control group, as seen in Figure 9(a). Masson's trichrome staining confirmed the findings from HE staining, revealing the higher osteogenic potential of Cry2 elevated cells (Figure 9(b)). Furthermore, immunohistochemistry revealed that OC, one of the most important osteogenic indicators, was increased in the CRY2-cDNA group (Figure 9(c)). Finally, our findings imply that upregulation of CRY2 promotes bone growth in vivo.

### 4.4. Upregulation of CRY2 Activated the Canonical WNT/*β*-Catenin Signaling Pathway

We investigated variations in the expression levels of the canonical WNT/*β*-catenin signaling to figure out how CRY2 governs osteoblast development and proliferation.

CRY2 overexpression promotes the WNT/*β*-catenin signaling pathway (Legend of the pathway during development, the conserved Wnt/-catenin pathway controls stem cell pluripotency and cell fate choices. Within distinct cell types and tissues, this developmental cascade integrates signals from other pathways such as retinoic acid, FGF, TGF, and BMP), as illustrated in Figure 10. More notably, we gathered and analyzed protein samples at 0 days, 7 days, 14 days, and 21 days after osteogenic induction and discovered that -catenin, the primary component in WNT/*β*-catenin signaling, was not only extremely represented in the CRY2-cDNA group at all 4-time points, accurate across the 2 tissue lines.

## 5. Conclusion

Rapid breakthroughs in biomedical technology have opened up hitherto unexplored fields of bone study. We have learned a lot about the various “origins” of osteoblast at the time of embryonic and postnatal lives. Recognizing the transcription and environment signals of osteogenesis is important for bone preservation and osteoprogenitor tissue migration during healing. According to the findings, CRY2 plays an important role in the ossification of mouse osteoblasts. CRY2's osteogenic regulatory activity is dependent on WNT/-catenin. This new function of CRY2 opens up new therapeutic possibilities, such as tissue engineering that uses CRY2 to enhance bone growth in bone deformities under rigorous self-healing circumstances. Anyhow, more in vivo and in vitro studies are required to confirm the practicality and medical use of CRY2 in treating bone abnormalities and also to uncover the precise molecular process of CRY2 in controlling osteoblasts.

## Figures and Tables

**Figure 1:** Schematic depiction of the methodology used.

**Figure 2:** Western blot assessment of CRY2 expressions in shRNAs consistently transfected tissues.

**Figure 3:** qRT-PCR was conducted to identify the expression degrees of OCN, ALP, Col1a1, and Runx2 in shRNA consistently transfected cells and regulation cells. (a) C3H10. (b) C2C12.

**Figure 4:** AR and ALP staining in CRY2 shRNA consistently transfected tissues contrasted with control cells.

**Figure 5:** AR staining was measured at 562 nm. (a) C3H10. (b) C2C12.

**Figure 6:** Relative ALP activity estimated during osteoblast differentiation. (a) C3H10. (b) C2C12.

**Figure 7:** The mRNA degrees of CRY2 identified by RT-qPCR in miR-7-5p upregulation tissues.

**Figure 8:** Measurement of OCN in tissues transfected with miR-7-5p only or miR-7-5p plus CRY2 cDNA by RT-qPCR.

**Figure 9:** Upregulation of CRY2 enhances osteoblast differentiation in vivo. (a) CRY2 overexpression enhanced bone-like pattern in vivo as identified by HE staining, (b) Masson's trichrome staining displayed equivalent pattern with HE staining, and (c) IHC staining for OC.

**Figure 10:** CRY2 upregulation enhances WNT/*β*-catenin activation.

## Data Availability

The data that support the finding of this study are available from the corresponding upon reasonable request.

## References

[1] Berger M. B., Cohen D. J., Olivares-Navarrete R. (2018). Human osteoblasts exhibit sexual dimorphism in their response to estrogen on microstructured titanium surfaces. *Biology of Sex Differences*.

[2] Narayanan A., Srinaath N., Rohini M., Selvamurugan N. (2019). Regulation of Runx2 by microRNAs in osteoblast differentiation. *Life Sciences*.

[3] Liu B., Lu Y., Wang Y., Ge L., Zhai N., Han J. (2019). A protocol for isolation and identification and comparative characterization of primary osteoblasts from mouse and rat calvaria. *Cell and Tissue Banking*.

[4] Gomathi K., Akshaya N., Srinaath N., Moorthi A., Selvamurugan N. (2020). Regulation of Runx2 by post-translational modifications in osteoblast differentiation. *Life Sciences*.

[5] Garg P., Mazur M. M., Buck A. C., Wandtke M. E., Liu J., Ebraheim N. A. (2017). Prospective review of mesenchymal stem cells differentiation into osteoblasts. *Orthopaedic Surgery*.

[6] Mammoli F., Castiglioni S., Parenti S. (2019). Magnesium is a key regulator of the balance between osteoclast and osteoblast differentiation in the presence of vitamin D3. *International Journal of Molecular Sciences*.

[7] Zhang Y., Gu X., Li D., Cai L., Xu Q. (2020). METTL3 regulates osteoblast differentiation and inflammatory response via Smad signaling and MAPK signaling. *International Journal of Molecular Sciences*.

[8] Tang Z., Xu T., Li Y., Fei W., Yang G., Hong Y. (2020). Inhibition of CRY2 by STAT3/miRNA-7-5p promotes osteoblast differentiation through upregulation of CLOCK/BMAL1/P300 expression. *Molecular Therapy-Nucleic Acids*.

[9] Kim K., Kim J. H., Kim I., Seong S., Kim N. (2020). Rev-erb*α* negatively regulates osteoclast and osteoblast differentiation through p 38 MAPK signaling pathway. *Molecules and Cells*.

[10] Hirai T. (2018). Regulation of clock genes by adrenergic receptor signaling in osteoblasts. *Neurochemical Research*.

[11] Karsenty G. (2020). Transcriptional control of osteoblast differentiation and function. *Principles of Bone Biology*.

[12] Takarada T., Xu C., Ochi H. (2017). Bone resorption is regulated by circadian clock in osteoblasts. *Journal of Bone and Mineral Research*.

[13] Chan W. C. W., Tan Z., To M. K. T., Chan D. (2021). Regulation and role of transcription factors in osteogenesis. *International Journal of Molecular Sciences*.

[14] Peng F., Shi J., Cai W., Zhou S., Zhang Y. (2018). Cryptochrome 1 promotes low-level laser irradiation-induced bone marrow mesenchymal stem cells proliferation and differentiation. *Journal of Biomaterials and Tissue Engineering*.

[15] Zheng J., Zhang L., Tan Z. (2021). Bmal 1-and Per 2-Mediated Regulation of the Osteogenic Differentiation and Proliferation of Mouse BMSCs by Modulating the Wnt/*β*-Catenin Pathway. *Molecular Biology Reports*.

[16] Luo B., Zhou X., Tang Q. (2021). Circadian rhythms affect bone reconstruction by regulating bone energy metabolism. *Journal of Translational Medicine*.

[17] Min H. Y., Jang W. G. (2017). Circadian clock gene per 1 mediates BMP2-induced osteoblast differentiation in MC3T3-E1 cells. *Journal of Life Science*.

[18] Pauly K. L. (2020). *The effects of electromagnetic wave stimulation (EMS) on osteoblast differentiation and activity (Doctoral dissertation), [Ph.D. thesis]*.

[19] Wu Q. Y., Wang J., Tong X. (2019). Emerging role of circadian rhythm in bone remodeling. *Journal of Molecular Medicine*.

[20] Tsang K., Liu H., Yang Y., Charles J. F., Ermann J. (2019). Defective circadian control in mesenchymal cells reduces adult bone mass in mice by promoting osteoclast function. *Bone*.

[21] Zhuo H., Wang Y., Zhao Q. (2018). The interaction between Bmal 1 and per 2 in mouse BMSC osteogenic differentiation. *Stem cells international*.

[22] Maria S., Witt-Enderby P. A. (2017). Circadian regulation of bone. *Circadian Rhythms and Their Impact on Aging*.

[23] Li H., Zhou L., Sun S. (2021). *Cholesterol 25-Hydroxylase Promotes Osteogenesis and Suppresses Adipogenesis of Bone Marrow Stromal Cells via mTOR Signaling Pathway*.

[24] Karvande A., Kushwaha P., Ahmad N. (2018). Glucose dependent miR-451a expression contributes to parathyroid hormone mediated osteoblast differentiation. *Bone*.

[25] Yin C., Tian Y., Yu Y. (2019). A novel long noncoding RNA AK016739 inhibits osteoblast differentiation and bone formation. *Journal of cellular physiology*.

[26] Paine A., Woeller C. F., Zhang H. (2018). Thy1 is a positive regulator of osteoblast differentiation and modulates bone homeostasis in obese mice. *The FASEB Journal*.

[27] Bao Q., Chen S., Qin H. (2017). Constitutive *β*-catenin activation in osteoblasts impairs terminal osteoblast differentiation and bone quality. *Experimental Cell Research*.

